# A Prospective Study of Using Chaihu Shugan Powder Combined with *Zu San Li* Acupoint Stimulation to Improve the Prognosis of Liver Stagnation and Qi Stagnation Syndrome in Acute Pancreatitis

This article has been retracted.

**DOI:** 10.1155/2022/3177201

**Published:** 2022-11-04

**Authors:** Wei-Wei Lu, Xiao-Yan Duan, Jian-Li Ni, Sheng-Liang Zhu, Ai-Hua Fei, Xiao-Su Wang

**Affiliations:** ^1^Department of Gastroenterology, Yueyang Hospital of Integrated Traditional Chinese and Western Medicine, Shanghai University of Traditional Chinese Medicine, Shanghai, China; ^2^Department of General Practice, Xinhua Hospital, Shanghai Jiaotong University School of Medicine, Shanghai, China; ^3^Department of Gastroenterology, Xinhua Hospital, Shanghai Jiaotong University School of Medicine, Shanghai, China; ^4^Department of Traditional Chinese Medicine, Xinhua Hospital Chongming Branch, Shanghai, China; ^5^Department of Traditional Chinese Medicine of Xinhua Hospital, Shanghai Jiao Tong University School of Medicine, Shanghai, China

## Abstract

**Background:**

This study aimed to explore the clinical efficacy of Chaihu Shugan powder combined with *Zu San Li* acupoint stimulation on the acute pancreatitis of liver and qi stagnation syndromes, the protection of intestinal barrier function, the prevention of severe tendency, and safety evaluation.

**Method:**

Data were collected from October 2019–June 2021 at Xinhua Hospital, which is affiliated with Shanghai Jiao Tong University School of Medicine, Emergency Department. Eighty patients with acute pancreatitis were randomly divided into a control treatment group (40 people) and a combined traditional Chinese medicine (TCM) treatment group (40 people). Detailed records of hospitalised patients were obtained, including the general situation of patients' clinical diagnosis and clinical examination before and after treatment. The changes in inflammatory and immune indexes before and after treatment were recorded.

**Result:**

Compared with the standard treatment group, the relief time of abdominal pain in the TCM treatment group was significantly shortened with statistically significant differences. Compared with the standard treatment group, the levels of WBC, ALT, CA, hemodiastase, lipase, TG, and other factors in the TCM treatment group decreased, whereas the levels of DB, SCR, cholesterol, K^+^, and other factors increased. The differences were statistically significant (*P* < 0.05).

**Conclusion:**

Chaihu Shugan powder combined with *Zu San Li* acupoint stimulation can reduce the clinical manifestations of liver and qi stagnation syndromes of acute pancreatitis, protect the intestinal barrier function, prevent the tendency of severe illness and improve the prognosis.

## 1. Introduction

Acute pancreatitis (severe acute pancreatitis, SAP) is an inflammatory disease of the pancreas that is characterised by rapid onset and rapid change and often induces systemic and local complications. Dangerous and complicated conditions and high mortality have been found in 20%–30% of patients [1]. Acute pancreatitis (AP) is among the most common acute abdominal diseases. AP is clinically characterised by local inflammation of the pancreas with or without changes in other organ functions. It is also characterised by rapid and variable disease progression. At present, it is unclear why some patients experience severe pancreatitis [2]. A multicentre prospective study of patients with acute pancreatitis reported a mortality rate of 17% [3]. Although the overall mortality rate for all hospitalised patients with acute pancreatitis was approximately 10% (2%–22%), the mortality rate for patients with severe acute pancreatitis can reach 30% [4]. This not only consumes plenty of health resources but also results in serious social and economic burden.

The Chaihu Shugan powder from Jing Yue Book regulates the liver and qi acupuncture therapy and has the characteristics of Chinese medicine. *Zu San Li* point is one of the main acupoints with the function of regulating the spleen and stomach, supplementing qi, channelling channels, activating collaterals, and dispersing weather and dampness. Intestinal barrier dysfunction in patients with acute pancreatitis can lead to bacterial migration and cause systemic inflammatory response syndrome, leading to acute exacerbation of the disease. Therefore, improving intestinal barrier function, inhibiting systemic inflammatory response syndrome, and preventing and treating acute exacerbation is the key to controlling disease progression [5–7].

This prospective study used Chaihu Shugan powder combined with *Zu San Li* acupoint stimulation to improve the prognosis of liver and Qi stagnation syndromes in acute pancreatitis. The clinical efficacy of these treatments in terms of protecting intestinal barrier function and preventing severe tendency in the safety evaluation was investigated.

## 2. Method

### 2.1. Inclusion Criteria

① The diagnosis of acute pancreatitis was revised according to the international consensus of Atlanta Classification and Definition in 2012 and was in line with the diagnostic criteria of liver and qi stagnation syndromes in the consensus of integrated Chinese and Western Medicine for acute pancreatitis diagnosis and treatment in 2017. ② Regardless of gender, patients aged between 18 and 85 years old and their guardians agreed to participate in the study and signed informed consent.

### 2.2. Exclusion Criteria

① The patient did not meet the diagnostic criteria of liver and qi stagnation syndromes of acute pancreatitis. ② The patient joined other clinical trials 3 months before the onset. ③ The patient was under 18 years old or over 85 years old. ④ Severe onset of the disease required surgery and other nonmedical treatment. ⑤ Patients with mental illness, severe liver and kidney failure, severe cardiovascular and cerebrovascular diseases, and patients with advanced tumors were excluded.

### 2.3. Elimination Criteria and Discontinuation Criteria

① Poor compliance and inability to adhere to treatment or quit without any reason were reasons for elimination. ② Patients with serious adverse reactions or complications did not continue with the treatments.

According to the relevant literature review, the standard deviation of the CAT score of the two groups was assumed to be 7. The test boundary was set as 3. The test efficacy was 80%, and alpha = 0.05. According to the sample size calculation formula proposed by Chow for the efficiency test, the minimum sample size to be calculated was 34. Considering the 15% shedding rate, 40 people in each group were required.

#### 2.3.1. Standard Treatment Group (Control Group)

In accordance with the principle of internal medicine comprehensive treatment of acute pancreatitis treatment, the following treatments were administered. A fast continuous gastrointestinal decompression on fluid resuscitation (when necessary), provision of acid suppression inhibitory enzyme antibiotics (when necessary), and enteral nutrition parenteral nutrition (when necessary) were performed to maintain water and electrolyte balance rehydration therapy. Regular oral rhubarb and mirabilite topical routine important treatments were also administered. Early use of ventilators in patients with acute respiratory distress syndrome (ARDS) and hemofiltration in patients with acute renal failure (RF) was performed.

#### 2.3.2. Chinese Medicine Treatment Group (Treatment Group)

Eighty patients were randomly divided into control and traditional Chinese medicine treatment groups according to random number table standards. Two groups were calculated by the conventional treatment of acute pancreatitis diagnosis and treatment. The traditional Chinese medicine treatment group was administered Chaihu Shugan powder at 100 ml each time three times a day and 5 days. At the same time, in the *Zu San Li* acupoint acupuncture points, the following were conducted. Piercing was performed at 1.5 inches with a filiform needle, and the needle was retained for 30 min. This was done once a day for 5 days. The clinical indicators were measured and compared with those before treatment and with those of the control treatment group.

#### 2.3.3. Detection of Clinical Efficacy and Clinical Indicators of TCM before and after Medication

Curative effect evaluation of TCM syndromes: TCM syndromes of patients were recorded.

Evaluation of clinical symptoms and signs: The patients were evaluated immediately after admission, and the patients who met the inclusion criteria were given medication within 24 h after evaluation. The APACHE score was recorded for observation, and the relief time of abdominal pain and abdominal distension was recorded in both groups. The entire process is shown in Figure 1.

Results of the laboratory examination efficacy evaluation: Peripheral blood routine and CRP amylase lipase liver function, blood lipid, blood glucose, electrolyte, plasma endotoxin, blood calcium, PCT, and other inflammatory factors should be performed before and after admission for treatment. The effects of Chaihu Shugan powder combined with acupoint stimulation on systemic inflammatory response and relief time of abdominal pain and abdominal distension were observed.

The SPSS 19.0 statistical software was used for processing. Measurement data were expressed as mean standard deviation (*x* ± *s*). *T*-test was used for comparison between the two groups, and a nonparametric rank-sum test was used for data with uneven variance. For the data obtained from multiple measurements of the same observation index of the same patient at different time points, ANOVA of repeated measurement data was used. *P* < 0.05 was considered statistically significant.

## 3. Result

In the basic information description of the patients in the control group and the treatment group, the mean plus or minus standard deviation of age in the control group was 49.4 ± 17.6, and that in the treatment group was 52.9 ± 18.9. The male/female ratio in the control group was 26/14, and that in the treatment group was 25/15.

APACHE II, as a scoring system that includes multiple factors, can make a quantitative evaluation of the patient's condition and estimate the overall situation of the patient from an overall perspective. It can be seen that the basic situation of patients in the two groups was the same, which excluded the influence of these basic factors on the follow-up study and ensured the consistency of the subsequent experimental conditions. Make further preparations for the follow-up experiment.

The length of stay in the hospital of the control group was 7.9 ± 2.6, and that of the treatment group was 9.5 ± 4.3. The APACHE II score of the control group was 3.6 ± 2.2, whereas that in the treatment group was 3.4 ± 2.4. Traditional Chinese medicine syndrome in the control group was 4.9 ± 2.8, and this was 5.3 ± 2.9 in the treatment group (Table 1).

In terms of the number of TCM symptoms, the treatment group selected patients with more severe TCM symptoms than the control group, which was also reflected in the length of hospital stay. It is convenient for a more objective and obvious comparison of subsequent experimental results.

The abdominal pain relief time between the two groups was 74.4 ± 22.8 in the control group and 33.3 ± 11.5 in the treatment group, and the difference was statistically significant (*P* < 0.05). There was a significant difference in abdominal pain relief time.

In the changes in blood test indexes in the two groups, the decrease in the indexes of PCT, AST, TB, and BUN in the treatment group did not reach statistical significance, and the decrease in the indexes of WBC, ALT, and CA in the treatment group was more obvious in statistical significance compared with the control group. CRP and neutrophilic granulocyte percentage (N%) are not of statistical significance between the two groups. Among the increased indicators, the DB and SCR in the treatment group increased but were not as obvious as those in the control group (Table 2). The patient responded well and positively to the treatment, as can be seen from the significant decline in white blood cells.

Among other clinical indicators, hemodiastase, lipase, TG, and blood glucose values decreased more significantly in the treatment group than in the control group. The amylopsin and blood lactic acid in the treatment group did not decrease significantly. Cholesterol and Ca^2+^ in the control group increased more obviously in statistical significance, and endotoxin indexes are not of statistical significance in both groups (Table 3). Compared with the control group, the blood lipids in the experimental group decreased significantly, reflecting the therapeutic effect of the experimental group.

## 4. Discussion

Acute pancreatitis is a common clinical acute abdomen, which is a pathophysiological process with both systemic reactions and local lesions. Although most patients with acute pancreatitis showed slight symptoms, the prognosis was good, but 20%–30% of the patients showed severe complications, such as necrosis or organ failure, with an AP total mortality of 5%–10% [8].

At present, the research status of TCM in acute pancreatitis shows that TCM plays an important role in the treatment of acute pancreatitis (AP), including the effectiveness of various therapeutic methods such as traditional Chinese medicine gavage, enema, external application of TCM, intravenous drip, acupuncture, and so on [9, 10].

Application of traditional Chinese medicine in the early stage of the disease can help relieve clinical symptoms and signs, reduce complications, and reduce mortality [11], indicating that traditional Chinese medicine can improve intestinal function, regulate immune function, and improve blood circulation by reducing the level of inflammatory factors so as to block the progress of inflammation and play a therapeutic role [12].

In the treatment of severe acute pancreatitis, we should follow the principle of the stage of the disease, use the methods of using the method of simple Chinese medicine and acupuncture, and treat the blood stasis and the form of the blood stasis [13, 14]. We completed a prospective study using Chaihu Shugan powder combined with Zu San Li acupoint stimulation to improve the prognosis of liver stagnation and Qi Stagnation syndrome in acute pancreatitis. In order to expand ideas for the prevention and treatment of acute pancreatitis.

At present, no good treatment method is available to address clinical to acute pancreatitis patient' systemic inflammation reaction and the underlying cause, namely, intestinal barrier function disorder. According to traditional medicine, liver stagnation and qi stagnation are important early signs of the pathogenesis of acute pancreatitis; thus, the treatment of acute pancreatitis by addressing liver stagnation and qi stagnation has positive significance [15]. The main mechanism of rapid progression of the disease is closely related to the production and release of inflammatory transmitters [16]. Pancreatic cell damage can occur for a variety of reasons, starting with a local inflammatory response that releases inflammatory transmitters into the bloodstream; it activates white blood cells, thereby causing an inflammatory cascade and systemic inflammatory response syndrome (SIRS); rapid deterioration and progression to multiple organ dysfunction syndromes (MODS) occurs [17].

Research scholar Wilmore [18] proposed the central organ theory of intestinal disease; that is, intestinal dysfunction may be an important factor that causes SIRS and MODS. Normal intestinal mucosa can play its barrier function and effectively prevent approximately 40 trillion bacteria. Endotoxin transfers out of the intestinal lumen, thereby blocking the translocation of bacterial toxins in the intestinal lumen and preventing damage to the body [19]. Intestinal organs are a hub of MODS; therefore, they are inflammatory transmitter extenders [20].

According to the basic clinical conditions of the two groups, the age and length of hospital stay of patients with Traditional Chinese Medicine (TCM) syndromes in the treatment group were higher than those in the control group, indicating that the basic conditions of patients before enrolment were worse. However, the results were better in terms of the time to abdominal pain relief and other measures that followed. Scientists have been discussing acupuncture [21]. Acupuncture treatment is being studied in a growing number of diseases and experiments on different species [22–24]. Using Zu San Li acupuncture to treat acute pancreatitis is a part of acupuncture therapy in Chinese medicine, which is the characteristic therapy of Chinese medicine. It is performed in accordance with the theory of TCM syndrome differentiation to treat acute pancreatitis [25–27].

Table 2 shows that the abdominal pain relief time of the treatment group was significantly shorter than that of the control group. Firstly, the pain of patients was reduced, suggesting that TCM compound therapy for acute pancreatitis may play a therapeutic role from different angles and through different targets. A large number of clinical and basic studies have not only confirmed the therapeutic effect of Chinese herbal formulas on acute pancreatitis but also preliminarily revealed the mechanism of these therapeutic effects [28, 29]. Sometimes, fatal acute pancreatitis is caused by a systemic uncontrolled inflammatory response, and the resulting gastrointestinal function damage is one of the main causes of death. Effective maintenance of gastrointestinal function can improve the prognosis of acute pancreatitis [30].

As shown in Table 2, the levels of WBC, ALT, and CA factors in the TCM treatment group were all reduced, which indicated a better treatment effect in the treatment group compared with the control group. In the indexes of PCT, CRP, N%, and BUN, the decrease or increase in the degree of the two groups were almost the same. In the indexes of AST and TB, the decreasing extent of the treatment group was less than that of the control group, which may be caused by different underlying diseases. In DB and SCR, the increase in the treated group was not as high as that in the control group, which may be related to the important mode of action. The levels of lipase, TG, and other factors decreased, as shown in Table 3. Those in the control group also decreased, but not as much as those in the treatment group. In particular, the decrease in lipase was very significant. The cholesterol and K^+^ factor levels in the treatment group increased. The elevation of cholesterol was not as high as that of the control group, but the elevation of K^+^ level exceeded that of the control group. In amylopsin, the decline was slightly greater in the control group than in the treatment group. There was little difference between the levels of blood glucose, Ca^2+^, endotoxin, and blood lactic acid, and thus, these can be ignored.

This study provided a more detailed scientific basis for the active development of traditional Chinese medicine and the promotion of the application of the method of regulating the liver and regulating qi combined with acupuncture therapy in preventing acute pancreatitis from becoming severe, which has high medical value and social significance [31]. At the same time, this study also had some shortcomings. Firstly, the experimental sample size was not large enough. The experimental sample size needs to be expanded. Secondly, there were fewer experiments for reference. Thirdly, the principle underlying the specific mechanism of TCM required further experimental research for clarification.

## 5. Conclusion

Chaihu Shugan powder combined with Zu San Li acupoint stimulation can improve the intestinal barrier function of clinical symptoms of liver and qi stagnation syndromes of acute pancreatitis. This also improved the prognosis. This treatment can be considered as a clinical intervention for patients with pancreatitis complicated by severe infection.

## Figures and Tables

**Figure 1:** Flowchart of inclusion and exclusion criteria for the entire experiment.

**Table 1:** Clinical Profile of SAP Patients at admission in two groups. TCM: traditional Chinese Medicine; APACHE II: acute physiology and chronic health evaluation II. The data are presented as the mean plus or minus the mean.

Characteristics	Control (*n* = 40)	Treatment (*n* = 40)
Age (year, ±s)	49.4 ± 17.6	52.9 ± 18.9
Gender (case, M/F)	26/14	25/15
Hospital days (day, ±s)	7.9 ± 2.6	9.5 ± 4.3
APACHE II (score, ±s)	3.6 ± 2.2	3.4 ± 2.4
Traditional Chinese medicine (TCM) syndromes (num, ±s)	4.9 ± 2.8	5.3 ± 2.9

**Table 2:** Blood index fluctuation of SAP Patients in two groups.

Item	Control (*n* = 40)	Treatment (*n* = 40)	*t* value	*P*
Relief time of abdominalgia (hours, ±*s*)	74.4 ± 22.8	33.3 ± 11.5	−3.34	<0.05
PCT	−0.4	−0.1	2.113	<0.05
CRP	−30.0	−30.0	4.352	0.043
WBC	−3.6	−5.3	7.644	0.034
N%	−16.5	−16.5	8.987	0.028
ALT	−25.9	−27.3	2.619	0.068
AST	−23.05	−22.7	1.078	0.098
TB	−8.7	−6.4	12.454	0.014
DB	+2.2	+0.5	8.140	0.034
BUN	−0.9	−0.8	1.989	0.060
CA	−37.3	−40.8	2.544	<0.05
SCR	+12.6	+3.8	2.019	0.051

PCT: procalcitonin (ng/mL); CRP, C-reactive protein (mg/L); WBC, white blood cells (10^9/L); N%, neutrophilic granulocyte percentage; ALT, alanine aminotransferase (u/L); AST, aspartate aminotransferase (u/L); TB, total bilirubin (*μ*mol/L); DB, direct bilirubin (*μ*mol/L); BUN, blood urea nitrogen (*μ*mol/L); CA, carbonic anhydrase (u/ml); SCR, serum creatinine (umol/L). The difference sign indicates the change in the mean before and after treatment (−: up, +: down). *P* < 0.05 indicates the presence of a significant difference between the two groups.

**Table 3:** Clinical test items of SAP patients in two groups.

Item	Control (*n* = 40)	Treatment (*n* = 40)	*t* value	*P*
Haemodiastase	−282.4	−365.6	7.452	0.037
Amylopsin	−88.1	−78.1	7.988	0.030
Lipase	−685.0	−1372.2	1.095	0.098
TG	−4.3	−8.3	12.011	0.015
Cholesterol	+0.8	+0.3	2.009	0.051
Blood glucose	0.0	−0.2	2.013	0.073
K^+^	0.0	+4.9	9.693	0.025
Ca^2+^	+0.4	0.0	1.263	0.081
Endotoxin	0.0	0.0	^*∗*^	^*∗*^
Blood lactic acid	−0.4	−0.2	18.986	0.016

Haemodiastase (U/L); amylopsin (U/L); Lipase (U/L); TG, triglyceride(mmol/L); cholesterol (mmol/L); blood glucose (mmol/L); K^+^, potassium (mmol/L); Ca^+^, calcium (mmol/L); endotoxin (EU/mg); blood lactic acid (mmol/L). All values are mean values in fluctuation. The difference sign indicates the change in the mean before and after treatment (−: up, +: down); ^*∗*^ Endotoxin showed no change; thus, there was no point in comparing it with others. *P* < 0.05 indicated a significant difference between the two groups. The above differences were statistically significant (*P* < 0.05).

## Data Availability

All data are collected from October 2019 to June 2021 at Xinhua Hospital affiliated with Shanghai Jiao Tong University school of medicine, the emergency department of the standard of 80 patients with acute pancreatitis. The data is stored in the electronic case system of Xinhua Hospital。
